The article "Analysis of the Diagnostic Efficacy of DOTATATE Imaging Combined with CGA and BSP Detection Mode for NEN Patients with Bone Metastasis" was retracted in 2023. Reasons: signs of a paper mill; compromised peer review; unreliable results or conclusions.

# Analysis of the Diagnostic Efficacy of DOTATATE Imaging Combined with CGA and BSP Detection Mode for NEN Patients with Bone Metastasis

**DOI:** 10.1155/2022/6279826

**Published:** 2022-07-23

**Authors:** Lei Lei, Tao Du, Jianbo Yang, Liang Cai, Huipan Liu, Yue Chen

**Affiliations:** ^1^Department of Nuclear Medicine, Affiliated Hospital of Southwest Medical University, Luzhou 266427, China; ^2^Nuclear Medicine and Molecular Imaging Key Laboratory of Sichuan Province, Luzhou 266427, China; ^3^Institute of Nuclear Medicine, Southwest Medical University, Luzhou 266427, China

## Abstract

In order to explore the clinical efficacy of DOTATATE imaging combined with CGA and BSP in the diagnosis of bone metastasis in patients with NENs, a total of 100 NEN patients treated in our hospital from January 2021 to January 2022 were analyzed. All patients are divided into bone metastasis group and nonmetastasis group according to pathological examination results. The differences of DOTATATE imaging, CGA, and BSP are compared, and ROC curves are obtained to analyze the clinical efficacy of the three indicators in single application and combined diagnosis. The results show that AUC, sensitivity, and specificity of DOTATATE, BSP, and CGA combined diagnosis are higher than those of single diagnosis (*P* < 0.05). It is clearly evident that DOTATATE test, BSP, and CGA can obtain accurate results in the diagnosis of bone metastasis in NEN patients, and those combined diagnosis can improve the diagnostic efficiency.

## 1. Introduction

Neuroendocrine tumors (NENs) mainly originate from neuroendocrine cells and are common in digestive organs, such as gastrointestinal tract, pancreas, and lung organs. After the occurrence of the disease, the abnormal increase of neuramines and peptides will cause a variety of clinical symptoms. However, there are no typical symptoms in the early stage of the disease. When the group reaction occurs, some patients will be in progress. Therefore, exploring an effective diagnostic scheme has important guiding significance for disease evaluation and treatment [1]. According to whether the tumor has hormone secretion function and whether there are clinical symptoms caused by hormones, neuroendocrine tumors are divided into two categories: nonfunctional (about 80%) and functional (about 20%). Nonfunctional gastrointestinal and pancreatic neuroendocrine tumors mainly show nonspecific gastrointestinal symptoms or local tumor occupying symptoms, such as progressive dysphagia, abdominal pain, abdominal distension, diarrhea, abdominal mass, jaundice, or melena. Functional gastrointestinal and pancreatic neuroendocrine tumors are mainly characterized by clinical symptoms caused by biologically active hormones secreted by the tumor, such as skin flushing, sweating, asthma, diarrhea, hypoglycemia, refractory peptic ulcer, and diabetes. Functional gastrointestinal and pancreatic neuroendocrine tumors are mainly pancreatic neuroendocrine tumors, including insulinoma, somatostatin tumor, glucagon tumor, and gastrinoma. High expression of somatostatin receptor (SSTR) is the main feature of NENs. The long-term prognosis of most patients is poor, and the diagnostic effect of conventional imaging techniques will be unable to achieve the expected result. Tetraazacyclododecane-1, 4, 7, 10-tetraacetic acid-D-phenylalanine 1-tyrosine 3-threonine 8-octreotide (1, 4, 7, 10-tetraazacyclododecane-n, N, N) N-tetraacetic acid-D-Phe1-Tyr3-Thr8-octreotate (DOTATATE) is the preferred diagnostic technique for clinical overexpression of SST, with advantages of fast imaging and high spatial resolution [2, 3]. Chromogranin A (CGA) and bone sialoprotein (BSP) are clinical markers for the diagnosis of tumors with high sensitivity [4, 5]. At present, there are few studies on the clinical efficacy of DOTATATE, BSP, and CGA in diagnosing bone metastasis of NENs. The purpose of this study is to analyze the clinical value of DOTATATE, BSP, and CGA in the diagnosis of bone metastasis in NENs and to provide data support for the follow-up diagnosis and treatment of bone metastasis in NENs.

This paper is organized as follows: Section 2 discusses the related work.  Section 3 is the proposed methods and observation indicators.  Section 4 is the experimental results and comparative analysis. Finally, in Section 5, some concluding remarks are made.

## 2. Related Work

Bone is rich in capillaries and blood transport. Accordingly, the probability of tumor metastasis is very high. Clinically, common CT, MRI, and PET/CT detection schemes can obtain relatively accurate diagnosis results. Previous studies believe that bone metastasis of NENs is a rare condition. Reasonable and accurate comprehensive diagnosis has important guiding significance for the clinical evaluation of bone metastasis in NEN patients and the optimization of treatment plan [6, 7].

Some research results show that the SUVmax of patients with bone metastasis was significantly higher than that of patients without bone metastasis. The imaging technology can accurately diagnose early NEN bone involvement and asymptomatic bone metastasis, and the detection sensitivity is >90.00% [8]. Besides, the patients with NEN bone metastasis will have higher SUVmax value. It also further suggests that DOTATATE examination technology has certain application value in NEN bone metastasis. By analyzing the main mechanism, the bone is affected by physiological factors and takes relatively little DOTATATE, which lays a good foundation for image examination of bone metastatic lesions [9]. PET phenomenon cannot accurately detect small diameter lesions, while CT can make up for this deficiency. However, CT has a low spatial resolution [10]. PET/CT examination using DOTATATE technology can realize the image complementarity of the two impact tests. Comprehensive diagnosis can be made based on DOTATATE uptake characteristics of lesions, precise positioning, and high-resolution morphological change images, thus effectively improving sensitivity and specificity and enabling clinicians to make accurate clinical judgment [11, 12]. There are still false positive and false negative results of DOTATATE, which may be caused by the high expression of SSTR in both inflammatory activated macrophages and lymphocytes, leading to an increase in the intake of imaging agent, resulting in false positive [13].

Chen et al. [14] pointed out that CGA is mainly distributed in chromaffin granules of endocrine cells and is abnormally expressed in many endocrine tumors. It is a common marker in clinical tumor diagnosis and is related to bone metastasis of tumor cells [15]. For patients with bone metastases, there is a high level of CGA. It is speculated that the mechanism may be that CGA is a hydrophilic secretory protein with acidic characteristics. As a part of neuropeptide family, the protein is widely distributed in neuroendocrine tumors in neuroendocrine tissues and is not expressed in non-NEN patients. Therefore, NENs can be accurately diagnosed. With the aggravation of the disease of the tumor, the abnormal increase of bone metastasis occurred in patients [16]. BSP acid glycoprotein is a kind of exist in the matrix, to participate in the trabecular bone, osteoblast combined process is involved in and plays an important role, and the existing research indicates that BSP high expression of bone metastases in breast cancer and is a sign of poor prognosis in patients with tumor; the research results show that the group of patients with bone metastasis BSP level is obviously higher, consistent with previous studies [17]. Analysis of the mechanism is mainly promoting blood vessel growth effects of BSP, integrin in physiological or pathological condition of angiogenic endothelial cells abnormally elevated; the BSP is the best ligands of integrin, and the interaction between tumor cells and bone cells in the bone microenvironment is crucial to the development of metastasis [18].

## 3. Proposed Methods and Observation Indicators

A total of 100 NEN patients treated in our hospital from January 2021 to January 2022 are selected as the research subjects, the male-to-female ratio was 45/55, the age was 32-79 years old, with an average of 50.34 ± 10.22 years old, and the cases of pancreas, rectum, lung, thymus, and thyroid are 25 cases, 27 cases, 22 cases, 13 cases, and 13 cases, respectively. There are 23 patients in G1 phase, 35 in G2 phase, and 42 in G3 phase. According to pathological examination results, they are divided into bone metastasis group and nonmetastasis group, 40 cases and 60 cases, respectively. Inclusion criteria are as follows: (1) NEN was confirmed by clinical laboratory examination and pathological examination [19], (2) clinical suspicion of bone metastasis, (3) clearly study all operations and matters needing attention and sign informed consent voluntarily, and (4) no long-acting radionuclide labeled SSA treatment was received within 1 month before the examination. Exclusion criteria are as follows: (1) history of other malignant tumors; (2) incomplete clinical data; (3) short-acting octreotide was taken within 24 h before DOTATATE examination, and long-acting octreotide was taken within 1 month before DOTATATE examination; and (4) DOTATATE test contraindications. This study should be in accordance with the criteria of the Declaration of Helsinki and has been approved by the medical Ethics Committee of our hospital.

### 3.1. BSP and CGA Detection Methods

Rabbit anti-human BSP, CGA monoclonal antibody and DAB kits, hematoxylin, and second antibody (horseradish peroxide labeled) are purchased from Abcam, Zhongshan Jinqiao, and Santa Cruz. The tumor tissue is continuously sliced into 4 *μ*m thick slices and baked at 65°C for 2 h. Immunohistochemical PV-9000 two-step detection is performed on 100 tumor samples of the study subjects strictly according to the kit instructions to observe the expression of BSP and CGA.

### 3.2. DOTATATE Imaging Detection Method

During the phase of drug preparation, the generator (itG GE-68/GA-68 generator) was given 4 mL HCL at a concentration of 0.05 mol/L one day before 68GA-DOTATATE labeling. 130 *μ*L 1 mol/L sodium acetate and 20 *μ*g DOTATATE dissolved in 20 *μ*L high pure water were added into the reaction tube before labeling. The generator was cleaned with 2 mL HCL at a concentration of 0.05 mol/L, and the waste liquid was poured out. Subsequently, 2 mL × 0.05 mol/L HCL leaching CA-68 was added into the reaction tube. Under the reaction condition of 90°C and 10 min, the cooled sealed reaction tube was diluted evenly with 10 mL water, and the Vac C-18 column was washed with 10 mL water after passing through the mixture. The product was washed with ethanol (0.5 mL), and 5 mL water for injection was given to the column. Finally, the injection was obtained through a sterile filter membrane.

Specific requirements for PET/CT examination include as follows: the patient is advised to take 4-6 h fasting and rest quietly for 10-15 min. 68Ga-DOTATATE is intravenously injected for 3-5 mCi and rested quietly for 45-50 min. The trunk of 5-bed is collected by Siemens Biograph, Germany. Model 64 PET/CT (tube current, tube voltage, rotation time, pitch, and layer thickness of 100 mAs, 120 kV, 0.5 s, and 0.9 and 5 mm, respectively) is performed. CT images are used for PET attenuation correction. PET (3D emission acquisition, 3 min/bed) is updated to an iterative method of point diffusion technique (TureX). The correction conditions are 172 mm × 172 mm image matrix, 21 subsets, 3 iterations, and 4 mm half-width Gaussian filtering and increased scattering.

PET/CT image results are analyzed by 2 physicians with senior professional titles in our hospital, without informing the doctor of the patient's pathological grade. According to the absorption degree of 68Ga-DOTATATE, the lesions can be divided into the following levels: (1) zero absorption of imaging agent was 0. (2) The imaging agent was slightly absorbed, and the mediastinal blood pool > absorption level was grade 1. (3) The medium absorption of imaging agent and liver physiological level ≥ absorption level > mediastinal blood pool was grade 2. (4) The imaging agent was ingested in large quantities, and the liver < absorption level was 3. All bone metastases were expressed as semiquantitative maximum standard uptake value (SUVmax) and region of interest (ROI) profiles around the lesion, and ROI profiles selected by SUVmax were calculated by computer.

### 3.3. Observation Indicators

In this study, the observation indicators include as follows: (1) SUVmax data of DOTATATE test for metastatic and nonmetastatic NEN patients are recorded and compared; (2) BSP and CGA data of patients with and without metastasis were recorded and compared; (3) using pathological examination as the gold standard, the detection and accuracy of DOTATATE test, BSP, and CGA in the diagnosis of bone metastasis in NEN patients are calculated. The criteria for the positive expression of BSP and CGA are brownish yellow granules in tumor cell cytoplasm. The sections are observed by two physicians with senior professional titles in our hospital. The scores of 10 representative sections with high magnification field of vision (×400) were averaged, and the difference of observation results between the two physicians was no more than 3 points. Percentage score of positive cells is as follows: 0 score without positive cells. Positive cells accounted for 1%-10% of 1 point. Positive cells accounted for 11%-50%, 2 points. Positive cells accounted for 51% ~80%, 3 points. Positive cells accounted for 81% ~100%, 4 points. Staining intensity score of positive cells are as follows: negative was 0; weak positive score is 1; moderately positive is 2 points; strong positive is 3 points. DOTATATE imaging criteria should adhere to the following principles: (1) the positive criteria were that the metabolism of normal liver tissue is lower than that on PET images observed by the naked eyes; (2) negative or positive diagnosis of lesions should be discussed together if there is no agreement; (3) draw receiver operating characteristic curve (ROC curve) to analyze the diagnostic value of single application and combined application of DOTATATE examination, BSP, and CGA in NEN bone metastasis.

The software SPSS 22.0 is employed to carry out effective processing of the data and test the normality of the measurement data. The normal distribution of the measurement data is presented in the form of $\overset{¯}{x}\pm s$, *t*-test is adopted, and % is used to represent the count data, and *x*^2^ test is performed, *P* < 0.05, and the difference was statistically significant.

## 4. Experimental Results and Comparative Analysis

### 4.1. Differences between Transferred and Untransferred SUVmax Data

The SUVmax of the metastatic group is significantly higher than that of the nonmetastatic group, and the difference is statistically significant (*P* < 0.05), as shown in Table 1 and Figure 1.

### 4.2. Differences between BSP and CGA Proteins with and without Metastasis

The protein expression levels of BSP and CGA in the metastatic group are significantly higher than those in the nonmetastatic group, and the differences are statistically significant (*P* < 0.05), as shown in Table 2 and Figure 2.

### 4.3. Detection of DOTATATE, BSP, and CGA Bone Metastases

DOTATATE can detect 7 false positive cases and 4 false negative cases of NEN bone metastasis, 7 false positive cases and 3 false negative cases of BSP, and 8 false positive cases and 3 false negative cases of CGA. Three combined diagnoses are false positive in 1 case and 2 cases.  Table 3 demonstrates the results of DOTATATE diagnosis of NEN bone metastasis, and Table 4 shows BSP diagnosis results of NEN bone metastasis. In Table 5, CGA results of NEN bone metastasis can be observed. In addition, the results of DOTATATE, BSP, and CGA combined diagnosis of NEN bone metastasis are illustrated in Table 6 in detail. NEN patients are the high-risk group of bone metastasis, and relevant research shows that the proportion of bone metastasis in NEN patients is 4.00%-15.00%. Among the 100 subjects included in this study, 40 cases are found to have bone metastasis, accounting for 40.00%, which is significantly different from the data reported. Analysis of the reasons may be that most of the patients included in this study are in advanced stage of disease at the time of diagnosis. Thus, the risk of bone metastasis is high.

### 4.4. Effectiveness of DOTATATE, BSP, and CGA in Diagnosing NEN Bone Metastasis

AUC of DOTATATE, BSP, and CGA alone and combined diagnosis of NEN bone metastasis are all >0.75, and sensitivity and specificity are all greater than 80.00%. AUC, sensitivity, and specificity of DOTATATE, BSP, and CGA alone and combined diagnosis are all higher than that of single diagnosis, and the differences were statistically significant (*P* < 0.05), as shown in Table 7 and Figure 3. Combined with ROC curve analysis of the above mechanism of action studies, the combined diagnosis of DOTATATE, BSP, and CGA as well as the separate diagnosis of each indicator has good clinical efficacy, suggesting that DOTATATE, BSP, and CGA can be used as evaluation indicators of bone metastasis in NEN patients, and the combined diagnosis can further improve the clinical diagnostic efficacy.

## 5. Conclusions and Future Work

In this study, the analysis of the diagnostic efficacy of DOTATATE imaging combined with CGA and BSP detection mode for NEN patients with bone metastasis is conducted. From the experimental results, it can be observed that the protein expression levels of SUVmax, BSP, and CGA in the metastatic group are higher than those in the nonmetastatic group (*P* < 0.05). The number of false positive cases of bone metastasis of NENs in DOTATATE, BSP, and CGA is 7, 7, and 8, respectively. The number of false negative cases is 4, 3, and 3, respectively. In addition, the false positive cases of the three combined diagnoses are 1 case and 2 cases, respectively. DOTATATE, BSP, and CGA are all abnormal elevated in patients with NEN bone metastasis. Accurate results can be obtained for the three separate diagnoses of NEN bone metastasis, and the three combined detection modes can effectively improve the diagnostic efficiency of NEN bone metastasis, which is worthy of promotion and application in clinical work of NEN bone metastasis. The limitations of this study are as follows: the design idea is not perfect, and the small sample size may increase the data bias. In addition, the differences between patients with bone metastases of different disease severity and other risk individuals need further study. In the future, we will analyze the relationship between disease and bone metastasis in detail to further consolidate the research results.

## Figures and Tables

**Figure 1:** SUVmax data changes between transferred and untransferred.

**Figure 2:** Changes of BSP and CGA proteins with and without metastasis.

**Figure 3:** ROC curve of NEN bone metastasis diagnosis of DOTATATE, BSP, and CGA.

**Table 1:** SUVmax data differences between transferred and untransferred ($\overset{¯}{x}\pm s$).

Group	SUVmax (nmol/L)
Transfer group (*n* = 40)	3.70 ± 1.12
No transfer group (*n* = 60)	1.72 ± 0.39
*t*	12.620
*P*	<0.001

**Table 2:** Differences of BSP and CGA proteins between metastatic and nonmetastatic groups ($\overset{¯}{x}\pm s$).

Group	BSP (nmol/L)	CGA
Transfer group (*n* = 40)	39.34 ± 11.66	9.34 ± 1.66
No transfer group (*n* = 60)	30.12 ± 9.89	6.12 ± 1.39
*t*	4.249	10.494
*P*	<0.001	<0.001

**Table 3:** Results of DOTATATE diagnosis of NEN bone metastasis.

DOTATATE	Pathology		Total
	Positive	Negative	
Positive	33	4	37
Negative	7	56	63
Amount to	40	60	100

**Table 4:** BSP diagnosis results of NEN bone metastasis.

BSP	Pathology		Total
	Positive	Negative	
Positive	33	3	36
Negative	7	57	64
Amount to	40	60	100

**Table 5:** CGA results of NEN bone metastasis.

CGA	Pathology		Total
	Positive	Negative	
Positive	32	3	35
Negative	8	57	65
Amount to	40	60	100

**Table 6:** Results of DOTATATE, BSP, and CGA combined diagnosis of NEN bone metastasis.

DOTATATE+BSP + CGA	Pathology		Total
	Positive	Negative	
Positive	39	2	41
Negative	1	58	59
Amount to	40	60	100

**Table 7:** Diagnostic efficacy of DOTATATE, BSP, and CGA for NEN bone metastasis.

Index	AUC	Standard error	Sensitivity	Specificity	*P*	95% CI
DOTATATE	0.879	0.040	91.20	93.30	82.50	0.801~0.958
BSP	0.888	0.039	89.70	95.00	82.50	0.811~0.964
CGA	0.875	0.041	88.40	95.00	80.00	0.794~0.956
DOTATATE+BSP + CGA	0.971	0.020	93.50	96.70	97.50	0.932~1.000

## Data Availability

The simulation experiment data used to support the findings of this study are available from the corresponding author upon request.
